The article "Quantitative Evaluation of Chronic Obstructive Pulmonary Disease and Risk Prediction of Acute Exacerbation by High-Resolution Computed Tomography" was retracted in 2023. Reasons: unreliable results or conclusions; concerns about the data; concerns about the peer review; concerns about the citations.

# Quantitative Evaluation of Chronic Obstructive Pulmonary Disease and Risk Prediction of Acute Exacerbation by High-Resolution Computed Tomography

**DOI:** 10.1155/2022/6015766

**Published:** 2022-07-12

**Authors:** Qifeng Hua, Guoping Chen, Yin Yang, Shaoyi Leng, Zhenzhen Zhao, Feng Bai, Xiaowei Hu, Liyan Qiu, Zhe Yu, Hongbin Zhang, Jiapei Shi, Qi Dai

**Affiliations:** ^1^Department of Radiology, Hwa Mei Hospital, University of Chinese Academy of Sciences, Ningbo, China; ^2^Department of Respiratory Medicine, Hwa Mei Hospital, University of Chinese Academy of Sciences, Ningbo, China

## Abstract

**Objective:**

It is imperative to popularize the tertiary prevention of chronic obstructive pulmonary disease (COPD) and to improve the diagnosis and treatment.

**Methods:**

COPD patients were divided into mild (*n* = 18), moderate (*n* = 20), severe (*n* = 24), and extremely severe (*n* = 22) groups for performing high-resolution computed tomography (HRCT) and pulmonary function test. Serum procalcitonin (PCT) and high-sensitivity C-reactive protein (hs-CRP) were detected, and the occurrence rate of acute exacerbation COPD (AECOPD) was recorded during a 12-months follow-up period.

**Results:**

With an increase in the severity grade, the HRCT indexes, including emphysema index (EI), 1st and 15th percentile of inspiratory attenuation distribution (Perc1 and Perc15), ratio of expiratory/inspiratory mean lung density (MLD_ex/in_) and lung volume (LV_ex/in_), and ratio of the wall thickness to the outer diameter of the lumen (TDR), as well as percentage of the wall area to the total cross-sectional area (WA%) were increased with a decreased change in relative lung volume with attenuation values between −860 and −950 HU (RVC_−860to −950_) and lumen area (*A*_i_). These were correlated with the ratio of forced expiratory volume in 1 sec (FEV1) over forced vital capacity (FVC) (FEV1/FVC), the percentage of FEV1 the predicted value (FEV1%), and ratio of residual volume to total lung volume (RV/TLC). Body mass index, MLD_ex/in_, FEV1%, FEV1/FVC, and PCT had a predictive value to AECOPD, with the combined AUC of 0.812.

**Conclusions:**

HRCT imaging effectively classifies the severity of COPD, which combined with BMI, PFT, and serum PCT can predict the risk of AECOPD.

## 1. Introduction

Chronic obstructive pulmonary disease (COPD), as a life-threatening pathology of the lung, is defined as a clinical syndrome characterized by chronic respiratory symptoms, structural pulmonary abnormalities, lung function impairment, or any combination of these [1]. With a world prevalence of 10.1%, COPD will rise from the sixth to the third cause of death in the world in 2020, which will further lead to 4.4 million death yearly by 2040 [2, 3]. COPD as a very heterogeneous disease still remains underdiagnosed, primarily because it usually is considered to be a disease of the elderly [3, 4]. Hence, it is imperative to popularize the tertiary prevention of COPD and improve the diagnosis and treatment.

The development of imaging, especially the widespread use of multi-slice high-resolution computed tomography (HRCT), can show the fine anatomy of the lungs at low radiation doses [5]. HRCT requires short breath-holding time and can determine the local pathological changes of the lungs before pulmonary function tests show that the lung function is normal or the symptoms of COPD appear [6, 7]. HRCT is an ideal method to study the phenotype of COPD. Through quantitative analysis of the dynamic changes in the respiratory biphasic pixel index, CT scanning at the end of deep inspiration and expiration can be used to evaluate the pulmonary function test (PFT) directly and objectively [8, 9]. In addition, the systemic inflammatory response is a key factor in the occurrence and development of COPD. It has a strong effect on the progression of COPD and the formation of complications [10, 11].

Procalcitonin (PCT), an inflammatory marker, has been found in the past to be increased only in systemic bacterial infections [12]. Recently, following improvements in the sensitivity of the detection methods and lowering the diagnostic threshold, PCT has been used for detecting localized bacterial infections [13]. The PCT value increases rapidly and with high sensitivity and specificity after 1–2 h of lower respiratory tract inflammation [14]. High-sensitivity C-reactive protein (hs-CRP) is a nonspecific acute-phase protein that is often used as a sensitive index of inflammation [15]. The hs-CRP index will increase within a few hours after inflammation and return to normal with inflammation regression [16], and its higher serum level was associated with three-year all-cause mortality of COPD [17]. Serum PCT and hs-CRP levels have been reported to be good predicted values for COPD, especially for acute exacerbation of COPD (AECOPD) [18, 19].

In this study, HRCT was used to quantitatively analyze the lung function and phenotype of COPD patients. To that end, we evaluated lung changes in COPD and analyzed the correlation between HRCT imaging and PFT in quantitative evaluation of lung function. We also predicted the diagnostic value of HRCT in acute exacerbation to better evaluate disease progression in patients.

## 2. Materials and Methods

### 2.1. Research Subjects

Eighty-four COPD patients confirmed by the Global Initiative for the Prevention and Treatment of COPD (GOLD) [20] were treated in our hospital from May 2020 to April 2021. Exclusion criteria were as follows: lung cancer patients, history of chest surgery, such as heart valve replacement and lung volume reduction surgery (LVRS), congenital thoracic deformity, thoracic deformity caused by pulmonary tuberculosis, large infected area of the lung, consolidation of the lung, bronchial asthma, active pulmonary tuberculosis, interstitial fibrosis of the lung, pleural thickening, and massive pleural effusion, and heart, liver, and kidney insufficiency diseases; patients with an ongoing AECOPD will not be included in the study. This project was approved by the hospital ethics committee, and all patients agreed to accept the examination with a signed informed consent.

### 2.2. Pulmonary Function Tests (PFTs)

PFT was performed using a Master Screen lung function instrument (Jaeger Company, Germany) by experienced respiratory doctors. The subjects were seated and rested for 10 min. The main indexes were as follows: (1) The ratio of forced expiratory volume in 1 sec (FEV1) over forced vital capacity (FVC) (FEV1/FVC). (2) The predicted percentage value of FEV1 (FEV1%); and (3) The ratio of residual volume to total lung volume (RV/TLC). The patients were then divided into four groups, including mild group (*n* = 18, FEV1/FVC <70% and FEV1 ≥ 80%), moderate group (*n* = 20, FEV1/FVC <70% and 50% ≤ FEV1 < 80%), severe group (*n* = 24, FEV1/FVC <70% and 30% ≤ FEV1 < 50%), and extremely severe group (*n* = 22, FEV1/FVC <70% and FEV1 < 30%, or FEV1 < 50% plus chronic respiratory failure) according to a previous study [1].

### 2.3. Serum PCT and Hs-CRP Determination Method

Fasting venous blood samples were obtained in the morning, which were centrifuged at 3,000 rpm. The serum was separated and sent to the laboratory for detection. The serum concentration of PCT (EHPCTX5) and hs-CRP (KHA0031) was determined by human ELISA kits (Thermo Fisher Scientific Co., Ltd., China) strictly in accordance with the instructions.

### 2.4. The 128-Slice Biphasic HRCT Examination Method

The patients hold their breath at the end of deep inspiration and expiration to cooperate closely with the 128 slice CT scanner (Siemens Somatom definition AS+) without using contrast media. All subjects were in the supine position, holding their heads with both hands for scanning. Scanning parameters were as follows: Tube voltage, 120 kV; tube current, 50 mAs; pitch, 1.4; and collimation width, 0.6 mm. The CT scan images were transmitted to a Syngo Multimodality Workplace for postprocessing automatic analysis. The measurement threshold was between −1024 and −400 HU, the left and right lungs were automatically delineated, and the trachea and left and right bronchi were segmented. Six lung regions (the upper left, middle left, lower left, right upper, right middle, and right lower lung region) were horizontally segmented at three horizontal levels, including the aortic arch, the tracheal carina, and the inferior pulmonary vein (IPV). Three-dimensional analysis was applied in a semiquantitative evaluation of whole lung function and a quantitative assessment of the small airway structure.

### 2.5. Quantitative Analysis of Parameters

The following quantitative parameters were determined, including (1) emphysema index (EI): the area below −950 HU in CT thin-slice images (≤2 mm) was defined as “emphysema;” in this study, EI was the percentage of less than −950 HU voxels in the whole lung. (2) Emphysema Perc1% and Perc15% measures (1^st^ and 15^th^ percentile of inspiratory attenuation distribution): the frequency distribution of pixel attenuation values in the lung area was displayed after analyzing the HRCT data at the end of deep inhalation; all attenuation values lower than −950 HU on a histogram were defined as emphysema. (3) The air retention was evaluated by the ratio of mean lung density (MLD_ex_/_in_) between the expiratory phase and inspiratory phase in inspiratory and expiratory biphasic scanning. (4) The change in expiratory phase and inspiratory phase attenuation area of −860 to −950 HU model was considered as the airflow limitation caused by small trachea remodeling. The air retention was evaluated by the change in relative lung volume with attenuation values between −860 and −950 HU (RVC_−860 to −950_). (5) The ratio of expiratory/inspiratory lung volume (LV_ex_/_in_). (6) Multiplanar reformation (MPR) method was used to reconstruct the cross-sectional images perpendicular to the long axis of bilateral segmental bronchi, with the window width of 1,000 HU and the window level of −500 HU. The ratio of the wall thickness to the outer diameter of the lumen (TDR) = thickness (T)/bronchial diameter (D), WA = extrabronchial area (*A*_o_)− lumen area (*A*_i_), the percentage of the wall area to the total cross-sectional area (WA%) = (WA/*A*_o_) × 100%. Each index was measured three times at different positions to gain an average value.

### 2.6. Follow-Up

COPD patients were followed for 12 months, the participants were asked to record worsening or new daily respiratory symptoms and attend for exacerbation visits if necessary. An exacerbation was defined as an increase in respiratory symptoms for two consecutive days, with at least one major symptom (dyspnea, sputum purulence, or sputum volume) plus either another major symptom or a minor symptom (wheeze, cold, sore throat, or cough). The first day of these increased symptoms was defined as the day of onset of the exacerbation.

### 2.7. Statistical Analysis

SPSS 22.0 software was used for the analyses. The *χ*^2^ test was used to analyse the enumeration data. For measurement data, Student's *t*-test was employed to compare differences in two groups, and ANOVA and LSD test was used to compare differences among three or more groups. The relationships among HRCT lung function parameters and PFT parameters was assessed by Pearson's test. The diagnostic level of an acute exacerbation risk of COPD was predicted by an area analysis under the ROC curve. A *P* value < 0.05 was statistically different.

## 3. Results

Differences of the HRCT lung function and PFT parameters among patients with different grades of COPD.

With an increase grade of severity, FEV1% and FEV1/FVC decreased gradually in COPD patients with increased RV/TLC (*P* < 0.05), but there was no difference in FEV1/FVC between mild and moderate patients (*P* > 0.05). Besides, the lung function indexes of HRCT were also correlated with the severity of COPD. With an increase in severity grade, EI, Perc1, Perc15, MLD_ex/in_, LV_ex/in_, TDR, and WA% also gradually increased (*P* < 0.05, while RVC −860 to −950 and Ai gradually decreased (*P* < 0.05, Table 1).

### 3.1. Correlations among HRCT Pulmonary Function Parameters and PFT Parameters

Perc1, Perc15, and Ai were positively correlated with FEV1% and FEV1/FVC and negatively correlated with RV/TLC; while RVC_−860 to −950_, MLD_ex/in_, TDR, and WA% were negatively correlated with FEV1% and FEV1/FVC and positively correlated with RV/TLC (*P* < 0.05). EI was significantly correlated with only FEV1% and FEV1/FVC (*P* < 0.05, Table 2).

### 3.2. Prediction Value of HRCT, PFT, and Serum Indicators to AECOPD

There were 43 cases with AECOPD during the follow-up, as shown in Table 3; there was no obvious difference in age, smoking history, EI, Perc1, Perc15, RVC_−860 to −950_, LV_ex/in_, TDR, WA%, *A*_i_, RV/TLC, and hs-CRP between the two groups (*P* > 0.05). However, there were significant differences in the body mass index (BMI), MLD_ex/in_, FEV1%, FEV1/FVC, and PCT (*P* < 0.05). Specifically, the scores of MLD_ex/in_ and PCT in AECOPD patients were increased, while BMI, FEV1%, and FEV1/FVC decreased. Five indicators with significant differences (MLD_ex/in_, PCT, BMI, FEV1%, and FEV1/FVC) between the two groups were used to predict AECOPD, as shown in Figure 1 and Table 4. All the five indicators had a predictive value to AECOPD (*P* < 0.05) and the area under the curve (AUC) of the combination of them was 0.812.

## 4. Discussion

COPD is recognized as a heterogeneous disease [21]. Researchers are increasingly interested in classifying the clinical and pathophysiological heterogeneity of COPD into different phenotypes, and the phenotype of COPD is defined as one or several disease characteristics [22]. On the one hand, these pathological characteristics are relevant to disease symptoms, aggravation, treatment response, disease progression rate, and mortality and can evaluate the prognosis of the disease [23]. On the other hand, they can reflect the differences among COPD patients, including differences in the prognosis and treatment schemes, which are conducive to guiding individualized treatment of the disease [4, 24].

The 2018 revision [20] of the Global Initiative for COPD (GOLD) jointly published by the National Institutes of Health (NIH) and the WHO suggests that the PFT method is simple, repeatable, and convenient for large-scale popularization. However, sex, age, BMI, susceptibility, and other indicators vary from person to person. Therefore, using the same threshold for different people will lead to certain errors in examination results. Because the diversity of the pathological changes of the small airway, lung parenchyma, and pulmonary vessels in COPD cannot be determined by FEV1 [21], finding more sensitive examination methods to evaluate changes in the lung structure and function is an urgent task in current research. As computer and medical software technologies have developed rapidly, imaging examinations can accurately and sensitively find lesions in the early stage of disease. This has obvious advantages in the early diagnosis, quantitative analysis, and prognosis evaluation of COPD [25]. Compared with ordinary CT, HRCT has many technical advantages, such as thin layer, high spatial resolution reconstruction algorithm, and a short scanning time. HRCT not only reflects changes in the local anatomical structure in early COPD, it can also measure the mean lung density (MLD), lung volume, and pixel index (PI) and quantify the changes in lung function by using special image postprocessing software [26]. It has gradually become a research hotspot for evaluating the condition of COPD by quantitative bronchial measurements [27]. Our results reflected that similar to PFT, HRCT-related and serum inflammation indicators were tied to the phenotypic classification of COPD patients. Especially TDR, WA%, and *A*_i_ gradually increased or decreased with an increased phenotypic classification of patients. While there were obvious differences among the phenotypic classifications of the COPD patients, these results indicate that HRCT have value in the quantitative assessment of COPD. Although there are many HRCT parameters significantly relevant to the indexes of PFT, we think that HRCT cannot completely replace PFT in the assessment of the pulmonary function of COPD patients. It is more likely to be used as an auxiliary tool to improve the accuracy of severity grading.

Afterward, we analyzed the diagnostic value of HRCT parameters, PFT parameters, and serum PCT in AECOPD. Tsai et al. [28] clarified that about 600,000 people are admitted to the emergency departments for AECOPD every year in the United States. AECOPD has become the third major reason for emergency treatment besides cardiovascular and cerebrovascular diseases. It affects patients' quality of life and disease progression, and it is also relevant to cardiovascular diseases and other complications, mortality, and hospitalization rate, which largely increases medical expenses. It is estimated that AECOPD accounts for about 70% of the total COPD medical expenses [29, 30]. An oxidation-antioxidation imbalance, a significant increase in the oxidative stress level, and a rise in inflammatory mediators are considered the main reasons for pulmonary vascular remodeling, incomplete reversible airflow restriction, and aggravation of infection symptoms [30]. We found that MLD_ex/in_ and PCT were increased in patients with AECOPD, while BMI, FEV1% and FEV1/FVC decreased. Among these indexes, BMI, MLD_ex/in_, FEV1%, FEV1/FVC, and PCT, all had a predictive value to AECOPD, and the AUC of the combined diagnosis reached 0.810. However, there still exist a few limitations: First, although there still exist a higher serum level of hs-CRP in AECOPD patients than the SCOPD one, it showed no significance. The reason for this phenomenon may be the small sample size. Second, except for PCT and hs-CRP, the joint monitoring of changes in other inflammatory indicators (e.g., IL family, TNF-*α*) of COPD patients can also effectively and accurately observe the disease and reduce the risk of an acute attack [31], which would be further explored in the future.

To sum up, HRCT imaging can effectively classify the phenotype of COPD. Combined with serum, PCT can predict the risk of acute exacerbation of COPD. However, the evaluation of the pulmonary function of patients cannot completely replace traditional PFT, and HRCT may be a crucial supplementary tool for the overall evaluation of COPD. For one thing, it helps to improve the quantitative diagnosis level and accuracy of the evaluation of the severity of COPD patients. For another, it is significant for predicting the risk of AECOPD and providing early intervention in clinical practice.

## Figures and Tables

**Figure 1:** The ROC of BMI, MLDex/in, FEV1%, FEV1/FVC, and PCT to predict AECOPD. Acute exacerbation of chronic obstructive pulmonary disease (AECOPD); ratio of forced expiratory volume in 1 sec (FEV1) over forced vital capacity (FVC) (FEV1/FVC); percentage of FEV1 the predicted value (FEV1%); ratio of expiratory/inspiratory mean lung density (MLDex/in); procalcitonin (PCT); Body mass index (BMI).

**Table 1:** Comparison of the HRCT lung function and PFT parameters in COPD patients with different severity.

Parameters	Mild group (*n* = 18)	Moderate group (*n* = 20)	Severe group (*n* = 24)	Extremely severe group (*n* = 22)	*F*	*P*
FEV1%	81.87 ± 15.24	69.14 ± 11.71^*∗*^	35.98 ± 8.19^*∗*^^#^	26.14 ± 7.71^*∗*^^#&^	121.96	<0.001
FEV1/FVC (%)	63.18 ± 10.91	58.01 ± 9.74	41.51 ± 7.01^*∗*^^#^	33.15 ± 7.72^*∗*^^#&^	51.61	<0.001
RV/TLC (%)	41.40 ± 8.73	51.08 ± 9.71^*∗*^	62.14 ± 8.55^*∗*^^#^	70.12 ± 9.12^*∗*^^#&^	38.89	<0.001
EI (%)	11.82 ± 12.85	11.07 ± 8.20	18.53 ± 11.73^#^	24.54 ± 13.30^*∗*^^#^	6.06	0.001
Perc1 (HU)	−977.12 ± 20.53	−977.70 ± 14.58	−980.73 ± 17.76	−991.53 ± 14.93^*∗*^^#&^	3.27	0.026
Perc15 (HU)	−938.10 ± 20.38	−937.88 ± 17.80	−947.69 ± 22.64	−957.79 ± 19.11^*∗*^^#^	4.56	0.005
RVC _−860to−950_ (%)	−33.02 ± 27.36	−34.35 ± 21.05	−10.88 ± 12.48^*∗*^^#^	−5.45 ± 10.60^*∗*^^#^	13.61	<0.001
MLD_ex/in_	0.88 ± 0.08	0.89 ± 0.05	0.94 ± 0.03^*∗*^^#^	0.96 ± 0.02^*∗*^^#^	13.17	<0.001
LVe_x/in_	0.61 ± 0.17	0.58 ± 0.06	0.72 ± 0.10^*∗*^^#^	0.79 ± 0.10^*∗*^^#&^	15.81	<0.001
TDR	0.19 ± 0.03	0.22 ± 0.04^*∗*^	0.25 ± 0.03^*∗*^^#^	0.32 ± 0.03^*∗*^^#&^	50.80	<0.001
WA%	62.49 ± 4.51	69.11 ± 4.50^*∗*^	77.93 ± 7.20^*∗*^^#^	86.89 ± 4.11^*∗*^^#&^	79.90	<0.001
*A*_i_ (cm^2^)	17.60 ± 4.88	14.89 ± 4.61^*∗*^	9.10 ± 3.24^*∗*^^#^	4.18 ± 1.93^*∗*^^#&^	51.99	<0.001

Ratio of forced expiratory volume in 1 sec (FEV1) over forced vital capacity (FVC) (FEV1/FVC); percentage of FEV1 the predicted value (FEV1%); ratio of residual volume to total lung volume (RV/TLC); emphysema index (EI); 1st and 15th percentile of inspiratory attenuation distribution (Perc1 and Perc15); ratio of expiratory/inspiratory mean lung density (MLD_ex/in_) and lung volume (LV_ex/in_); ratio of the wall thickness to the outer diameter of the lumen (TDR); percentage of the wall area to the total cross-sectional area (WA%); change in relative lung volume with attenuation values between −860 and −950 HU (RVC_−860 to −950_); lumen area (*A*_i_). ^*∗*^Compared with the mild group, *P* < 0.05; ^#^compared with the moderate group, *P* < 0.05; and ^&^compared with the severe group, *P* < 0.05.

**Table 2:** Correlations among HRCT pulmonary function parameters and PFT parameters.

Parameters	FEV1%		FEV1/FVC (%)		RV/TLC (%)	
	*r*	*P*	*r*	*P*	*r*	*P*
EI (%)	−0.343	0.001	−0.281	0.010	0.171	0.119
Perc1 (HU)	0.371	0.001	0.352	0.001	−0.307	0.005
Perc15 (HU)	0.333	0.002	0.307	0.005	−0.320	0.003
RVC_−860to−950_ (%)	−0.583	<0.001	−0.525	<0.001	0.490	<0.001
MLD_ex/in_	−0.525	<0.001	−0.564	<0.001	0.362	0.001
LV_ex/in_	−0.032	0.773	−0.075	0.497	0.007	0.949
TDR	−0.624	<0.001	−0.588	<0.001	0.591	<0.001
WA%	−0.698	<0.001	−0.642	<0.001	0.594	<0.001
*A*_i_ (cm2)	0.665	<0.001	0.642	<0.001	−0.562	<0.001

Ratio of forced expiratory volume in 1 sec (FEV1) over forced vital capacity (FVC) (FEV1/FVC); percentage of FEV1 the predicted value (FEV1%); ratio of residual volume to total lung volume (RV/TLC); emphysema index (EI); 1st and 15th percentile of inspiratory attenuation distribution (Perc1 and Perc15); ratio of expiratory/inspiratory mean lung density (MLD_ex/in_) and lung volume (LV_ex/in_); ratio of the wall thickness to the outer diameter of the lumen (TDR); percentage of the wall area to the total cross-sectional area (WA%); change in relative lung volume with attenuation values between −860 and −950 HU (RVC_−860to−950_); lumen area (*A*_i_).

**Table 3:** Comparison of HRCT, PFT, and serum indicators between SCOPD and AECOPD patients.

Parameters	SCOPD (*n* = 41)	AECOPD (*n* = 43)	*P*
Age (years)	64.80 ± 8.80	66.37 ± 8.54	0.410
BMI (kg/cm^2^)	22.97 ± 1.40	21.42 ± 1.32	≤0.001
History of smoking (years)	19.34 ± 9.58	19.79 ± 11.65	0.848
EI (%)	16.81 ± 11.87	18.54 ± 11.35	0.499
Perc1 (HU)	−981.56 ± 17.59	−982.54 ± 17.98	0.802
Perc15 (HU)	−945.42 ± 19.85	−946.44 ± 23.05	0.829
RVC_−860to−950_ (%)	−19.26 ± 24.48	−20.29 ± 20.06	0.834
MLD_ex/in_	0.91 ± 0.06	0.93 ± 0.05	0.021
LV_ex/in_	0.68 ± 0.15	0.69 ± 0.12	0.817
TDR	0.24 ± 0.05	0.26 ± 0.06	0.105
WA%	73.84 ± 10.42	75.85 ± 10.54	0.387
*A*_i_ (cm^2^)	11.99 ± 6.54	10.07 ± 6.05	0.165
FEV1%	57.60 ± 27.40	44.93 ± 21.10	0.020
FEV1/FVC (%)	51.74 ± 15.57	44.22 ± 13.21	0.019
RV/TLC (%)	55.31 ± 15.13	58.92 ± 12.53	0.237
PCT (*μ*g/L)	0.97 ± 0.68	1.27 ± 0.74	0.028
Hs-CRP (mg/L)	36.93 ± 17.23	41.96 ± 13.93	0.076

Acute exacerbation of chronic obstructive pulmonary disease (AECOPD); stable COPD (SCOPD); ratio of forced expiratory volume in 1 sec (FEV1) over forced vital capacity (FVC) (FEV1/FVC); percentage of FEV1 the predicted value (FEV1%); ratio of residual volume to total lung volume (RV/TLC); emphysema index (EI); 1st and 15th percentile of inspiratory attenuation distribution (Perc1 and Perc15); ratio of expiratory/inspiratory mean lung density (MLD_ex/in_) and lung volume (LV_ex/in_); ratio of the wall thickness to the outer diameter of the lumen (TDR); percentage of the wall area to the total cross-sectional area (WA%); change in relative lung volume with attenuation values between −860and−950 HU (RVC_−860 to −950_); lumen area (*A*_i_); procalcitonin (PCT); high-sensitivity C-reactive protein (hs-CRP); body mass index (BMI).

**Table 4:** ROC analysis results.

Parameters	Cut-off value	Area	*P*	95% confidence interval (CI)		Sensitivity (%)	Sensitivity (%)
				Lower	Upper		
BMI	21.940	0.794	<0.001	0.698	0.891	69.77	78.05
MLD_ex/in_	0.925	0.645	0.022	0.526	0.764	58.54	72.09
FEV1%	59.745	0.631	0.038	0.511	0.752	74.42	53.66
FEV1/FVC (%)	46.515	0.653	0.015	0.535	0.771	67.44	63.41
PCT	0.775	0.639	0.028	0.520	0.758	58.54	67.44
Joint detection of 5 indexes	0.405	0.812	<0.001	0.719	0.905	68.29	88.37

Ratio of forced expiratory volume in 1 sec (FEV1) over forced vital capacity (FVC) (FEV1/FVC); percentage of FEV1 the predicted value (FEV1%); ratio of expiratory/inspiratory mean lung density (MLD_ex/in_); procalcitonin (PCT); body mass index (BMI).

## Data Availability

The data used to support the findings of this study are included within the article.
